This article has been retracted.

# miR-182-5p improves the viability, mitosis, migration, and invasion ability of human gastric cancer cells by down-regulating RAB27A

**DOI:** 10.1042/BSR20170136

**Published:** 2017-06-27

**Authors:** Yuling Li, Shudong Chen, Zhengfei Shan, Liyan Bi, Shengqiang Yu, Yongwei Li, Sen Xu

**Affiliations:** 1 Department of Pathophysiology, Binzhou Medical University, Yantai 264003, Shandong, China; 2 Department of Gastrointestinal Surgery Ward II, The Affiliated Yantai Yuhuangding Hospital of Qingdao University, Yantai 264000, Shandong, China; 3 Department of Urology, The Affiliated Yantai Yuhuangding Hospital of Qingdao University, Yantai 264000, Shandong, China; 4 Department of Transformative Otology and Neuroscience Center, Binzhou Medical University, Yantai 264003, Shandong, China; 5 Department of Biochemistry and Molecular Biology, Binzhou Medical University, Yantai 264003, Shandong, China

**Keywords:** gastric cancer, miR-182-5p, RAB27A

## Abstract

We investigated the effect of miR-182-5p on the viability, proliferation, invasion, and migration ability of human gastric cells by regulating the expression of RAB27A. Real-time PCR assay was used to detect the expression of miR-182-5 and RAB27A in human gastric carcinoma tissues, para-carcinoma tissues, and different cell lines. Western blotting was also used to determine the RAB27A expression in both tissues and cell lines. We chose the HGC-27 cell line as experiment subject as it demonstrated the highest miR-182-5p level. HGC-27 cells were transfected with different vectors and the cell viability, mitosis, invasion, and migration ability were measured through MTT assay, flow cytometry (FCM) analysis, Transwell assay, and wound healing assay. In comparison with the normal tissues, miR-182-5p is expressed at a higher level in gastric cancer (GC) tissues, while RAB27A is expressed at a lower level in cancerous tissues. The down-regulation of miR-182-5p and up-regulation of RAB27A can significantly decrease the viability, migration, invasion, and mitosis of HGC-27 cells. The target relationship between miR-182-5p and RAb27A was confirmed through a dual-luciferase reporter gene assay and Western blot assay. miR-182-5p enhances the viability, mitosis, migration, and invasion of human GC cells by down-regulating RAB27A.

## Introduction

Gastric cancer (GC) is one of the most common malignant tumors of the digestive system, has an estimated 951,600 new cases and causes 723,100 deaths every year [1]. Although there has been a steady decline in the incidence and mortality rate of GC in developed countries, in less developed areas, it still has a threatening third rank in both cancer incidence and mortality [1]. The causes for GC are complex and may include factors such as an unbalanced diet, smoking, alcohol, and infection of the *Helicobacter pylori* [2]. Furthermore, GC pathogenesis is also reported to be related with genetic factors such as DNA methylation, the epigenetic inactivation of several genes, gene amplifications and deletions, and aberrant somatic mutations [2].

The absence of specific clinical symptoms sets obstacles for the early diagnosis of GC [3]. Therefore, patients with GC are always diagnosed at advanced stages leading to serious metastasis and poor prognosis. The 5-year survival rate is less than 30% [4–6]. Surgery has been the primary treatment option for GC during the past few decades, with an auxiliary treatment of chemoradiation and chemotherapy [7,8]. Gene-based drug therapy is a potential approach for GC treatment [9]. However, due to the lack of understanding of the molecular mechanisms behind GC development, there is currently no effective therapy for GC [10].

RAB27A is an isoform of RAB27 and a member of the small GTPase Rab family. RAB27A is unique as its dysfunction is related to human hereditary diseases such as type 2 Griscelli syndrome [11]. Previous studies have reported that the deregulation of RAB27A is related with carcinogenesis and progressions such as colorectal carcinoma [12,13], pancreatic cancer [14], and lung cancer [15]. In breast cancer, the overexpression of RAB27A was found to promote various cell activities such as growth, invasion, and metastasis [16,17]. Additionally, scientists have found *in vivo* that RAB27A can serve as a prognostic biomarker in gliomas [18,19] and hepatocellular cancer [20]. All studies mentioned above jointly indicate that a close relationship exists between RAB27A and cancer. However, the role of RAB27A in GC has not been thoroughly explored. miRNAs are a collection of small non-coding RNAs with a length of 21–25 nt. Through binding to the 3′-UTR regions, miRNA can suppress gene expression at both the mRNA and translational levels [21,22]. Previous studies have suggested that miRNAs such as miR-29c, miR-135b, miR-193b, and miR-532-5p are key regulators of tumor proliferation, apoptosis, and migration. They can also serve as potential biomarkers and therapeutic targets in GC [23–25]. The aberrant expression of miR-182-5p has been proven to play an oncogenic role in variant malignant tumors such as bladder [26] and prostate cancer [27]. However, a study performed by Xu et al. [28] indicated that the down-regulation of miR-182-5p promotes the proliferation in renal cell carcinoma by targeting the AKT/FOXO3a signaling pathway.

Data from the TargetScan database suggest that a targeting relationship exists between miR-182-5p and RAB27A. We made the assumption that miR-182-5p regulates activity in GC cells by targeting RAB27A and conducted a series of experiments to test this hypothesis. We investigated the role of miR-182-5p and evaluated its regulatory mechanism in gastric tumorigenesis and progressions.

## Materials and methods

### Human tissues

Thirty human GC and the para-carcinoma tissues (the distance from the gastric carcinoma was 2 cm) were obtained from the Affiliated Yantai Yuhuangding Hospital of Qingdao University from March 20, 2015 to May, 20 2016. Samples were subsequently frozen in liquid nitrogen for further study. Para-carcinoma tissues were identified by three physicians in the hospital and confirmed to be cancer-free. All patients gave their informed consent and the ethical approval was obtained from the Human Ethics Committee of the Affiliated Yantai Yuhuangding Hospital of Qingdao University.

### Cell culture

Human gastric cancer (HGC) cell lines and human normal gastric cell lines comprising HGC-27, MKN-45, SGC-7901, and MGC-803 were bought from the cell bank of the Chinese Academy of Sciences (Shanghai, China) and cultured at the Roswell Park Memorial Institute (RPMI, New York, U.S.A.)-1640 with 10% fetal bovine serum (FBS) in a humidified atmosphere of 37°C and 5% CO_2_.

### RNA extraction and quantitative real-time PCR

Total RNA of tissues and cells were extracted using the TRIzol reagent according to the manufacturer’s instructions. Total RNAs (5 μg) and miRNAs (5 μg) were then reverse transcribed into complementary DNAs (cDNAs). The SYBR Green PCR mix was used for quantitative analysis in the quantitative real-time PCR (qRT-PCR) assay. The primers for miR-182-5p, *RAB27A*, and other genes were purchased from RiboBio Co., Guangzhou, China (Table 1). PCMV-Sport6 vectors (Invitrogen, Carlsbad, CA, U.S.A.) were used to recombine the RAB27A cDNAs, and DNA sequencing technique (contracted with Sangon Biotech, Shanghai, China) was used to confirm the successful recombination. U6 (RNU6B) and GAPDH were used as internal normalization standards for miR-182-5p and *RAB27A* mRNA respectively. Statistics were analyzed using the $2^{-\Delta \Delta C_{t}}$ method.

**Table 1:** Sequence of primers for the amplification of miRNA, RAB27A, and internal control genes

	Forward primer	Reverse primer
**miR-182-5p**	5′-TGCGGTTTGGCAATGGTAGAAC-3′	5′-CCAGTGCAGGGTCCGAGGT-3′
**U6**	5′-CTCGCTTCGGCAGCACA-3′	5′-AACGCTTCACGAATTTGCGT-3′
***RAB27A***	5′-GTAAGTGACATAGTAGTT-3′	5′-TTATTCGTAGGTCTAATG-3′
**GADPH**	5′-CCACCCAGAAGACTGTGGAT-3′	5′-TTCAGCTCAGGGATGACCTT-3′

### Cell transfection and grouping

To investigate the role of miR-182-5p on GC cell activities, HGC-27 cells in the logarithmic growth phase were transfected with 50 nM miR-182-5p mimics or 8 ng mimics control (GenePharma, Shanghai, China) using 1 μl of the Lipofectamine 2000 reagent. The groups were designed as follows: control group, miR-mimics group, anti-miR group, anti-negative control (NC) group, and miR-NC group. To study the role of *RAB27A* on GC cell activities, HGC-27 cells were transfected with lentiviral vectors recombined with human *RAB27A* gene sequence (the constructed vector was plenti-GIII-Ubc-*RAB27A*). These were assigned to the plenty-RAB27A group and cells transfected with the empty vector plasmid were designated as the NC group (named plenti-Null group).

### 3-(4,5-dimethylthiazol-2-yl)-2,5-diphenyltetrazolium bromide (MTT) assay

The viability of HGC-27 cells was measured using 3-(4,5-dimethylthiazol-2-yl)-2,5-diphenyltetrazolium bromide (MTT) assay. Cells were centrifuged and resuspended in the fresh complete medium. Subsequently, cells were seeded into 96-well plates with 1 × 10^4^ cells per well. After cells attached to the wall, cell viability was measured every 24 h. MTT solution (20 μl) and DMSO (150 μl) were added to cell culture and the absorbance rate of cells at 490 nm was measured using a microplate reader [29].

### Flow cytometry (FCM)

Cell cycle and cell apoptosis were assessed using flow cytometry (FCM) method. Forty eight hours after transfection, HGC-27 cells were washed with PBS and blended in a −20°C freezer with 70% alcohol at a concentration of 10^6^ cells/ml [29]. Subsequently, cells were left at 4°C overnight. On the next day, samples were centrifuged, washed with PBS, and then the supernatant was discarded. Cells were then resuspended in a liquor containing PI (50 mg/l) and RNase (50 mg/l) and incubated for approximately 25 min. In addition, other transfected cells were blended with the liquor Annexin V-FITC/PI according to the manufacturer’s instructions. After the cells were incubated for 20 min, FCM was used to assess cell apoptosis.

### Transwell assay

The invasion ability of cells was assessed using Transwell assay. The upper side of membranes was coated with Matrigel. RPMI 1640 (500 μl) containing 10% FBS was added to the lower chambers. Serum-free medium and the HGC-27 cells (3 × 10^5^) were placed in the upper chambers. After culturing for 48 h, 4% methanol and Crystal Violet were used to fix and stain the cells that invaded the membrane respectively. Subsequently, a microscope (100×) was utilized to count the cells in ten random fields in order to estimate the relative invasiveness of cells in different groups. Cell optical absorption was measured under 570 nm wavelength in each group.

### Wound healing assay

Wound healing assay was conducted to examine the migratory ability of HGC-27 cells. The cell suspension was seeded into a six-well plate with 2 ml of suspension in each well. After the confluence reached 80%, a sterile pipette was used to scratch the cell surface. Cells were then cultured in an incubator at 37°C and 5% CO_2_. The cell surface was photographed using an inverted microscope and the wound closure was measured at 0 and 24 h after scratching.

### Dual-luciferase reporter gene assay

The mutated *RAB27A* 3′-UTR was constructed using site mutation technology. The wild-type *RAB27A* 3′-UTR and mutated *RAB27A* 3′-UTR sequences were amplified using PCR. The amplified sequences were recombined with plasmids that contained the firefly luciferase gene. A total of 3 × 10^5^ cells were seeded into a 12-well plate and left overnight. When cells reached approximately 80% confluency, the [30] recombinant vectors and the Rellina Luciferase internal control pRL-CMV were co-transfected with either miR-mimics or miR-NC respectively into the HGC-27 cells using Lipofectamine 2000. The relative activity of luciferase was detected 48 h after transfection using the dual-luciferase reporter gene assay system according the manufacturer’s instructions.

### Western blotting

A total of 5 × 10^5^ cells were seeded into a 6-well plate, cultured overnight, and then the [30] total protein of tissues and cells was extracted using RIPA buffer. Subsequently, sodium dodecyl sulfate-polyacrylamide gel electrophoresis (SDS/PAGE; 12.5% gel) was conducted to isolate the proteins within the lysates. The proteins were then transferred onto a polyvinylidene difluoride (PVDF) membrane and 5% defatted milk was used to block the membrane at room temperature for 1 h. The membranes were incubated with primary antibodies overnight at 4°C. The next day, membranes were washed with tris-buffered saline with Tween (TBST) and incubated with horseradish peroxidase-coupled secondary antibodies. Signals were observed using chemiluminescence and the Western blotting detection system. ImageJ software was used to analyze the protein density.

### Statistical analysis

Statistical analysis was performed using SPSS 19.0 and GraphPad Prism 6.0 software. The statistical significance between two groups was determined using the Student’s test, and the mean calculated after each experiment was repeated three times. Measurement data are presented as the mean ± standard deviation ($\bar{x}\pm \text{s}$), and ANOVA was used to compare differences between multiple groups. A *P*-value < 0.05 is considered to be statistically significant.

## Results

### Overexpression of miR-182-5p in both GC tissues and cell lines

Quantitative real-time PCR analysis was utilized to investigate the expression of miR-182-5p in tissues and cells. The results demonstrated that GC tissues had a significantly higher expression of miR-182-5p than adjacent tissues (*P*<0.05) (Figure 1A). Moreover, the GC cell lines HGC-27, MKN-45, SGC-7901, and MGC-803 had higher levels of miR-182-5p than GES cell lines (Figure 1B). HGC-27 cells that had the highest level of miR-182-5p expression among the four GC cell lines were chosen for later studies.

**Figure 1:** miR-182-5p was overexpressed in GC tissues and cell lines; and RAB27A was low expressed in GC tissues (**A**) qRT-PCR analysis of relative miR-182-5p expression in GC tissues and cell lines. miR-182-5p showed a significantly higher expression in GC tissues than in adjacent tissues. ***P<0.001, statistically significant, compared with adjacent tissue. (**B**) HGC-27 cells expressed the highest level of miR-182-5p among the four GC cell lines. ***P<0.001, statistically significant, compared with GES cell line. (**C**) qRT-PCR analysis of the relative expression of RAB27A in GC and adjacent tissues. RAB27A mRNA was under expressed in GC tissues than in adjacent tissues. ***P<0.001, statistically significant, compared with adjacent tissue. (**D**) Western blot analysis on protein expression in GC and adjacent tissues. A lower level of RAB27A protein was seen in GC tissues than in adjacent tissues.

### Under expression of RAB27A in GC tissues

The RAB27A mRNA levels in GC and adjacent tissues were detected using qRT-PCR. We found that the expression of RAB27A mRNA in GC tissues was much lower than that in adjacent tissues (*P*<0.05) (Figure 1C). Western blotting assay was performed to determine the expression of RAB27A protein in GC and adjacent tissues. A lower level of RAB27A protein was seen in GC tissues in comparison with adjacent tissues (Figure 1D).

### Validation of RAB27A 3′-UTR as a direct target of miR-182-5p

The complimentary sequences of miR-182-5p and 3′-UTR of RAB27A were obtained from the TargetScan database and are shown in Figure 2(A). Luciferase assay was used to investigate the binding relationship between miR-182-5p and RAB27A. The wild-type and mutated *RAB27A* 3′-UTR segments were inserted into the plasmids and transformed into the pGLO-wt and pGLO-mut recombinant vectors. The recombinant vectors and the control plasmid pGLO-NULL were co-transfected with either miR-mimics or miR-NC in HGC-27 cells. The results showed a dramatic reduction in the luciferase activity of the miR-182-5p mimics + pGLO-RAB27A-3′-UTR (wt) group compared with the control group. This validates that RAB27A is negatively regulated by miR-182-5p (Figure 2B).

**Figure 2:** The targeting relationship between miR-182-5p and RAB27A (**A**) Schematic representation of binding site of miR-182-5p, the 3′-UTR sequence of RAB27A and the sequence of mutated RAB27A 3′-UTR. (**B**) The relative luciferase activity of the HGC-27 cells co-transfected with pGLO-wt, pGLO-mut as well as the pGLO-NULL with either miR-mimics or miR-NC respectively. Compared with the control group, only the luciferase activity in miR-182-5p mimics + pGLO-RAB27A -3′-UTR (wt) group was dramatically weakened, suggesting that RAB27A was negatively regulated by miR-182-5p; ***P<0.001, statistically significant, compared with miR-NC groups. (**C**) Western blot analysis of RAB27A protein levels in each group. Anti-miR group had the highest level of RAB27A protein among the three groups, indicating that the inhibition of miR-182-5p could increase the expression of RAB27A

Western blotting was used to determine the impact of anti-miR-182-5p on the expression of RAB27A (Figure 2C). RAB27A expression in the anti-miR, anti-NC, and control groups was detected and the results displayed that the inhibition of miR-182-5p could increase the expression of RAB27A.

### The viability of HGC-27 cells are repressed following the inhibition of miR-182-5p or the overexpression of RAB27A

Figure 3(A) shows that the viability of HGC-27 cells transfected with miR-182-5p inhibitors was significantly lower than the control and NC groups (*P*<0.01). A similar effect can be seen in the overexpression of RAB27A. Moreover, cells co-transfected with both miR-182-5p mimics and plenti-RAB27A showed no significant change in viability comparing with the control group. Collectively, the down-regulation of miR-182-5p or overexpression of RAB27A hinders the viability of HGC-27cells.

**Figure 3:** miR-182-5p down expression or RAB27A overexpression affected the viability, mitosis, and apoptosis of HGC-27 cells (**A**) MTT analyses showed the viability of HGC-27 cells. Compared with the control group and the anti-NC group, the viability of HGC-27cells transfected with anti-miR and plrnti-RAB27A was significantly lower than the anti-NC group and plenti-NULL group respectively. This illustrated that the down-regulation of miR-182-5p or overexpression of RAB27A hindered the viability of HGC-27cells. **P<0.01, compared with anti-NC group and plenti-NULL group. (**B** and**C**) FCM data showed the cell proportions in the G0/G1 phase in different groups. Compared with the corresponding NC group, both anti-miR and plenti-RAB27A groups showed a higher proportion of cells in the G0/G1 phase of HGC-27 cells. ***P<0.001 were considered statistically significant, compared with miR-NC and plenti-NULL groups respectively. (**D** and **E**) FCM analysis on the apoptosis rates of the HGC-27 cells 48 h after transfection. Compared with the anti-NC and plenty-NULL groups, the cell apoptosis dramatically increased in anti-miR and plenti-RAB27A groups. This indicated that the down-regulation of miR-182-5p or the up-regulation of RAB27A in HGC-27 cells may cause G0/G1 arrest and apoptosis.

### The inhibition of miR-182-5p or overexpression of RAB27A arrests cell cycle and promotes HGC-27 cell apoptosis

Figure 3 (B) and (C) suggests that there is no significant difference between the control and other NC groups. The proportion of HGC-27 cells in the G0/G1 phase increased in the anti-miR, plenti-*RAB27A* comparing with corresponding NC groups respectively (*P*<0.05). The proportion of HGC-27 cells in S-phase decreased in the anti-miR, plenty-RAB27A groups compared with corresponding NC groups respectively.

The apoptosis rates of cells in different groups are shown in Figure 3(D) and (E). There was no significant difference found between the control and all NC groups. Apoptosis cells in the anti-miR and plenti-RAB27A groups significantly outnumbered anti-NC and plenty-NULL groups (*P<*0.05). Collectively, G0/G1 arrest and apoptosis may be caused by anti-miR-182-5p or the overexpression of RAB27A in HGC-27 cells.

### The low expression of miR-182-5p or the overexpression of RAB27A suppresses the invasive and migratory ability of HGC-27 cells

No significant difference was seen between the control and other NC groups in regard to the invasive and migratory cell numbers. In order to explore the effect of miR-182-5p and RAB27A on cell invasiveness, we manipulated the expression of miR-182-5p and RAB27A in HGC-27 cells. The results are shown in Figure 4(A) and (B). We found that the number of cells that invaded the Transwell polycarbonate filter was significantly less in the anti-miR and plenti*-*RAB27A groups than in the anti-miR-NC and plenti-NULL groups (*P*<0.01). Moreover, there was little difference between the plenti*-*RAB27A+miR-mimics, control, plenti-NULL, and anti-miR-NC groups. These results demonstrate that the under expression of miR-182-5p or the overexpression of RAB27A can negatively regulate the invasiveness of HGC-27 cells.

**Figure 4:** miR-182-5p and RAB27A played a pivotal role in affecting the invasion and migration of HGC-27 cells (**A** and **B**) Transwell analysis of invasiveness of the transfected HGC-27 cells. Compared with the anti-miR-NC and plenti-NULL groups, there was little difference of the plenti-RAB27A+miR-mimics group, while fewer cells invaded through the membrane in the anti-miR and plenti-RAB27A groups. This result indicated that the under expression of miR-182-5p or overexpression of RAB27A could negatively regulate the invasiveness of HGC-27 cells. (**C**) The migratory abilities of cells in different transfection groups determined using wound healing assay. Compared with the corresponding NC groups, the migration of cells in the anti-miR group and plenti-RAB27A group significantly decreased. ***P<0.01 were considered statistically significant.

The migratory ability of HGC-27 cells was measured through the use of wound healing assay (Figure 4C). The figures show that the migration distance of cells in the anti-miR and plenti*-*RAB27A groups is significantly lower than that in the corresponding NC groups. The under expression of miR-182-5p or the overexpression of RAB27A can negatively regulate the migration of HGC-27 cells.

## Discussion

miR-182-5p was found to be overexpressed in GC tissues than in corresponding adjacent tissues. Similarly, miR-182-5p was found up-regulated in the four GC cell lines (HGC-27, MKN-45, SGC-7901, and MGC-803) in comparison with normal gastric epithelial cells (GES). These results suggest that miR-182-5p might be an oncogene of GC. Also, studies have demonstrated that miR-182-5p functions as an oncogene in different types of cancers such as melanoma [31] and breast cancer [32]. On the other hand, RAB27A was found to be down-regulated in GC tissues and cell lines, indicating that RAB27A may function as a tumor suppressor gene in GC. The Rab family reported by Grosshans et al. [33] was shown to play an essential role in membrane traffic by binding to their effectors. Scientists also found that Rab genes could regulates the activation of signal transduction, cell metabolism, membrane receptor, and the pathophysiology of diseases such as obesity, immune deficiency, diabetes, infection, and cancer [34]. This indicates a close relationship between Rab genes and diverse biological processes. RAB27A tends to be up-regulated in cancers such as hepatocellular carcinoma [20], breast cancer [16], and colorectal carcinoma [12]. In 2013, Wu et al. [35] found that RAB27A can enhance the glioma cell ability, accelerate proliferation and invasion, and inhibit cell apoptosis. We hypothesize that RAB27A may serve as a tumor suppressor by regulating signal transduction, cell metabolism, and membrane receptors in GC.

To see whether miR-182-5p function by regulating one of its effector gene RAB27A, we conducted dual-luciferase gene assay. miR-182 has been reported to target various tumor suppressors such as close homolog of LI (CHL1) and special AT-rich sequence-binding protein 2 (SATB2) in different cancers [36,37]. We confirmed that a targeting relationship exists between miR-182-5p and RAB27A. This was previously predicted by the TargetScan software. We speculate that the miR-182-5p/RAB27A axis has a close relationship with the formation and progression of GC.

It has been illustrated in previous studies that miR-182 and RAB27A are involved in regulating the biological process such as proliferation, apoptosis, migration, and invasion in various cancer cells [35,38,39]. In the present study, we observed that when miR-182-5p was inhibited or RAB27A was overexpressed, cell viability of GC cells line became inhibited, a large proportion of cells were held up in the G0/G1 phase, the apoptosis rate increased, and the invasive and migratory ability of GC cells were weakened. We demonstrated that miR-182-5p promotes the progression of GC by suppressing RAB27A. These may help understand how miR-182-5p/RAB27A influences GC progression at the cellular level.

In conclusion, the present study verifies that a negative regulatory relationship exists between miR-182-5p and RAB27A. This may be a novel target for the treatment and prognosis of GC and a possible diagnostic biomarker in clinical practice.

## Abbreviations

CHL1: close homolog of LI
FCM: flow cytometry
GC: gastric cancer
HGC: human gastric cancer
NC: negative control
qRT-PCR: quantitative real-time PCR
RPMI: Roswell Park Memorial Institute
SATB2: special AT-rich sequence-binding protein 2
